RETRACTED

# Analysis of Related Influencing Factors of Deep Vein Thrombosis after Lumbar Internal Fixation and Treatment Strategy

**DOI:** 10.1155/2021/9693012

**Published:** 2021-10-19

**Authors:** Sixiao Zhang, Guangjie Shen, Mingxing Luo, Xiqiang Zhong

**Affiliations:** ^1^Department of Orthopedics, Ningbo Hangzhou Bay Hospital, Ningbo, Zhejiang 315336, China; ^2^Department of Spinal Surgery, The Third Affiliated Hospital of Wenzhou Medical University, Ruian, Zhejiang 325000, China

## Abstract

Lumbar internal fixation is a traditional surgical method for the treatment of degenerative diseases of the lumbar spine. However, due to its large surgical trauma, it easily causes complications such as deep venous thrombosis (DVT) after the operation. DVT refers to the abnormal coagulation of blood in deep veins, blocking the lumen, causing venous blood return disorder, causing venous blood return disorder to cause swelling and pain, which affects the recovery of the patient's lumbar spine function. In severe cases, even complicated pulmonary embolism endangers the life and health of the patient. Therefore, it is extremely important to explore the related influencing factors and effective treatment of DVT. The purpose of this study was to investigate the influencing factors and effective treatment of DVT after lumbar internal fixation. Univariate analysis and multivariate a logistic regression model were used to analyze the related factors affecting DVT after lumbar internal fixation. Conventional treatments such as anticoagulation, promotion of venous blood return, and improvement of limb circulation were given to patients with DVT, and functional exercise was guided to compare the hypercoagulability and hyperviscosity of blood in patients with DVT before and after treatment. The results showed that the incidence of DVT after lumbar internal fixation was related to age, BMI, and bed time. Getting out of bed for functional exercise in time after surgery can effectively prevent the formation of DVT. Preoperative grading examination, intraoperative intervention, postoperative physical exercise, and other preventive guidance can be carried out according to different individuals during the perioperative period to prevent the formation of postoperative DVT.

## 1. Introduction

The lumbar spine is the hub of the movement of the human body's trunk and bears great pressure. With the increase of age, long-term involvement and excessive activity can easily lead to accelerated aging of the lumbar spine, leading to lumbar degenerative disease [1–3]. Lumbar internal fixation is a conventional surgical method for the treatment of degenerative lesions of the lumbar spine, but due to its large surgical trauma, it very easily causes complications such as deep venous thrombosis (DVT) after the operation [4–6]. DVT refers to the abnormal coagulation of blood in deep veins, blocking the lumen, leading to venous blood reflux disorder, resulting in venous blood reflux disorder causing swelling and pain, thus affecting the recovery of lumbar spine function of patients and even causing pulmonary embolism in severe cases endangering patients' life and health [7–10]. Therefore, it is extremely important to explore the relevant influencing factors and effective treatment methods for the formation of DVT. This study aims to explore the related factors and effective treatments of DVT after lumbar internal fixation. The detailed information is as follows.

RETRACTED

## 2. Materials and Methods

### 2.1. Patients

A total of 248 patients who underwent lumbar internal fixation in two hospitals from September 2017 to December 2019 were selected. Among them, there were 132 males and 116 females. The age ranged from 45 to 76 years, with an average age of (59.32 ± 7.29) years. All patients were examined by color Doppler ultrasonography of both the lower limbs after lumbar internal fixation and were divided into a DVT group (14 cases) and normal group (234 cases) according to whether they had DVT after operation. Diagnostic criteria for DVT [11, 12]: (1) the venous lumen cannot be compressed; (2) low echo or no echo in the lumen; (3) there was no blood flow signal, or only a few blood flow signals were detected in the vein of the thrombus segment; and (4) pulse Doppler showed no blood flow, or the spectrum did not change with respiration. Inclusion criteria: age >40 years; patients undergoing lumbar internal fixation in our hospital due to various lumbar diseases; all patients can tolerate the operation; preoperative Doppler ultrasound examination of both the lower limbs without DVT; and clinical data are complete. Exclusion criteria: patients with a history of lower limb arteriovenous diseases; patients with diseases affecting coagulation function; patients with serious cardiovascular and cerebrovascular diseases; people with cognitive function or mental disorder; cancer patients; patients with venous valve insufficiency of the lower extremities; patients with drug allergy; and patients with past history of cerebral infarction, pulmonary infarction, and venous embolism.

### 2.2. Treatment Methods

All DVT patients are given anticoagulation, to promote venous blood return and improve limb circulation, and other conventional treatments. Enoxaparin sodium 4000 IU for injection was given subcutaneously 12 h after surgery, once a day, for 2 weeks. Also, the patients were guided by functional exercise: straight leg raising exercise: the patients took the supine position and slowly raised one side of the lower limb after straightening the lower limbs until there was a sense of pulling pain and then raised the other side of the lower limb in the same way, 10 min/time. Hip and hip flexion exercise with both hands: the patient takes the lying position and then flexes the knee joint with both the hands and holds the knee to perform rhythmic hip flexion, and the lower limbs are alternately performed, 10 min/time. Ankle movement: ankle joint plantar flexion, dorsiflexion, and circular rotation are performed, each movement is repeated10 times and paused, 3s is maintained after each movement is in place, the feet are relaxed for 10 seconds between each movement, and each training is repeated 5 times. Double toe extension and flexion movement are performed, each movement is repeated 10 times, each movement is kept in place after stagnation and maintained for 3 s, the feet are relaxed 10 times between each movement, and each training is repeated 5 times.

RETRACTED

### 2.3. Observation Indicators

1. All patients' age, gender, body mass index (BMI), whether they smoke, drink alcohol, have complications such as hypertension, diabetes, and hyperlipidemia, and have intraoperative blood transfusion, operation time, bedtime, etc. were collected
2. Comparison of coagulation function: fasting venous blood was collected from DVT patients in the morning before and 14 days after treatment, and activated prothrombin time (PT), activated partial thromboplastin time (APTT), fibrinogen (FIB), and D-dimer (D-D) levels of DVT patients were detected by using an automatic hemagglutination apparatus
3. Comparison of hemorheology: the automatic hemorheology analyzer was used to detect the plasma viscosity, whole blood viscosity high-cut, low-cut, and hematocrit levels of DVT patients before and after treatment for 14 days

### 2.4. Statistical Methods

The results of this experiment were statistically analyzed by SPSS 20.0 (SPSS Co., Ltd., Chicago, USA). Count data were expressed by (rate), and the chi-square test was used for their comparison between groups. Measurement data were expressed by (mean ± standard deviation), and the *t*-test was used for their comparison between groups. Multivariate analysis adopts the multiple logistic regression model. *P* < 0.05 indicates that the difference is statistically significant.

## 3. Results

### 3.1. Single-Factor Analysis of DVT in Patients after Lumbar Internal Fixation

Univariate analysis showed that the patient's age, BMI, intraoperative blood transfusion, operation time, and bed time were all related to the occurrence of DVT after lumbar internal fixation (*P* < 0.05), as shown in Table 1.

RETRACTED

### 3.2. Multifactor Analysis of DVT in Patients after Lumbar Internal Fixation

Multivariate logistic analysis showed that age, BMI, and time in bed were independent influencing factors of DVT after lumbar internal fixation (*P* < 0.05), as shown in Tables 2 and 3.

### 3.3. Comparison of Coagulation Function before and after Treatment in Patients with DVT

After treatment, PT (16.84 ± 4.85)  s and APTT (29.69 ± 6.18)  s levels of DVT patients were higher than those before treatment, (12.82 ± 3.24) s and (26.43 ± 4.89)  s, and FIB (4.34 ± 1.08) g/L and D-D (0.64 ± 0.38) mg/L levels were lower than those before treatment, (7.24 ± 2.05) g/L and (1.16 ± 0.48) mg/L (*P* < 0.05), as shown in Figure 1.

### 3.4. Comparison of Hemorheology before and after Treatment in Patients with DVT

After treatment, DVT patients' plasma viscosity (1.38 ± 0.16) MPa·s, whole blood viscosity high-cut (5.02 ± 0.38) MPa·s, low-cut (9.08 ± 0.54) MPa·s, and hematocrit (43.23 ± 6.38)% were lower than those before treatment, (1.91 ± 0.24) MPa·s, (5.86 ± 0.45) MPa·s, (12.48 ± 0.73) MPa·s, and (52.15 ± 7.22)% (*P* < 0.05), as shown in Figure 2.

## 4. Discussion

DVT is one of the common diseases of the venous system. DVT can be seen in various main veins of the human body, but the most common site of occurrence is DVT in the lower limbs [13, 14]. Modern medicine believes that there are three basic factors in the formation of DVT, including blood flow stasis, vascular wall damage, and blood hypercoagulability [15]. Studies have shown that the following related factors can lead to the occurrence of DVT after lumbar internal fixation [16]: After prolonged bed rest or immobilization, the muscle pump function of the lower limbs is completely or partially lost, which affects venous return, and a large number of white blood cells accumulate and transfer to the damaged vascular intima, thereby activating the coagulation process; prolonged prone position during the operation may compress the inferior vena cava, iliac vein, and femoral vein, resulting in venous stasis of the lower extremities; lumbar spine fractures are often accompanied by spinal cord nerve injury or paralysis of the lower extremities, leading to dysregulation of the vena cava and lower extremity vascular nerves and the formation of DVT. Nicol et al. [17] pointed out that 50% of patients begin to develop DVT during surgery, and all individuals undergoing spinal surgery are high-risk patients with DVT. Those who do not have thrombosis can also develop chronic vascular disease, eventually leading to thrombosis. Therefore, it is the key to prevent the formation of DVT to start nursing work for patients as soon as possible after operation.

RETRACTED

There are many studies on the incidence of DVT after lumbar spine surgery, and the incidence is about 0.7%∼12.5%. DVT can cause other complications, such as pulmonary embolism, which can endanger the life of patients in severe cases [18]. Yang et al. [19] conducted a prospective study on the incidence of DVT in 710 patients undergoing single-level lumbar surgery and found that the incidence of DVT in lower limbs in 84 patients was 11.83%. Regression analysis found that advanced age, hypertension, and increased D-D were risk factors for DVT in lower limbs after surgery. Yoshioka et al. [20] prospectively observed the incidence of DVT after 459 cases of degenerative spine surgery and found that the incidence of DVT after cervical spine surgery was significantly lower than that after thoracolumbar surgery. The study also concluded that female, old age, surgical level, and impaired neurological function were all risk factors for DVT in lower limbs after spine surgery. Sebastian et al. [21] found the highest incidence of DVT after vertebrectomy (3.8%) and found that venous embolism after spinal surgery was associated with a longer hospital stay, concomitant cancer, high white blood cell count, paraplegia, low albumin, American College of Anesthesiologists grade 4 or above, higher body mass index, and longer operative time.

Our results showed that the patient's age, BMI, intraoperative blood transfusion, operation time, and bed time were all related to the occurrence of DVT after lumbar internal fixation. Multivariate logistic analysis showed that age, BMI, and time in bed were independent factors that affected patients with DVT after lumbar internal fixation. Older patients are more prone to thrombosis than younger patients due to the aging of the inner wall of the blood vessel and the change of blood vessel elasticity, the intima is rough and damaged, and most of them have other chronic diseases. Because of the high body fat in patients with high BMI, it is often easy to restrict the return of blood in the venous blood vessels, and the blood vessels are more likely to be damaged, leading to the formation of thrombus. Long-term bedridden patients have less activity, resulting in slower venous blood flow rate and increased viscosity, which in turn makes the patient more likely to develop thrombosis [22–24]. Also, the results of this study showed that, after treatment, the levels of PT and APTT in DVT patients were higher than those before treatment, and the levels of FIB, D-D, plasma viscosity, whole blood viscosity of high-cut, low-cut, and hematocrit were lower than those before treatment. It shows that postoperative anticoagulation for patients with DVT, promotion of venous blood return, improvement of limb circulation and other conventional treatments, and guiding them to perform functional exercises is beneficial to improve the patients' blood hypercoagulability and hyperviscosity. Slow venous blood flow, tube wall damage, and hypercoagulable state of blood are currently recognized as the three major pathological foundations of DVT. Lumbar internal fixation is one of the major orthopedic surgeries. Patients often need bed rest after surgery, and their venous blood flow is slowed down and hypercoagulable. Therefore, functional exercise guidance for patients after surgery is helpful to restore venous blood flow and relieve hypercoagulability.

RETRACTED

At present, DVT prevention measures after spinal fusion include basic prevention, mechanical prevention, and drug prevention. Basic prevention means that the patient actively or passively flexes and stretches the ankle and knee joints and keeps both the lower limbs above the level of the heart. The increased muscle contraction of the lower extremities makes the blood return rate of the lower extremities significantly faster than when the lower extremities are braked, which can reduce and prevent the formation of DVT in the lower extremities [25, 26]. Mechanical prevention refers to the use of various mechanical equipment to help patients contract the muscles of the lower limbs, speed up blood flow, and reduce the retention of blood in the veins of the lower limbs. These mechanical equipment mainly include grade elastic stockings, plantar pumps, and intermittent inflation and compression devices [27, 28]. At present, there is still controversy about whether to use drugs to prevent the formation of DVT after spinal surgery. Some scholars believe that the incidence of DVT after spinal surgery is low and there is no need for routine use of drugs for prevention. Currently, the most widely used anticoagulant drugs include low-molecular-weight heparin, rivaroxaban, aspirin, heparin, and warfarin. It has been reported that the formation of postoperative DVT after drug prophylaxis can significantly reduce the occurrence of DVT compared with mechanical prophylaxis or no other preventive measures [29, 30]. Low-molecular-weight heparin is widely used clinically and is one of the first-choice drugs to prevent the formation of DVT after surgery. It can significantly reduce the incidence of DVT after spinal surgery, and the risk of epidural hematoma and other bleeding events is low. Rivaroxaban is a new oral anticoagulant that is easy to use. Its effectiveness in preventing DVT formation after joint replacement has been confirmed, and its safety has obvious advantages over traditional anticoagulants [31, 32].

RETRACTED

Prevention of DVT should be carried out as soon as possible, and all patients should be classified according to the abovementioned risk factors before surgery. Patients with the abovementioned risk factors should be examined by relevant laboratory, and ultrasound examination of lower limbs should be performed if necessary, so as to timely understand the patient's hemorheology and lower limb blood vessels, and appropriate preventive treatment should be given. Because the patient needs to be in the prone position during the operation, the pressure of the abdominal vena cava will easily lead to blood stasis, which will form DVT, so the patient's position should be paid attention to during the operation to keep the abdomen suspended. Due to the relatively long spine surgery time, the surgery time should be shortened as much as possible during the operation, and the blood volume should be monitored to prevent insufficient blood storage. After the operation, the patient's eating habits should be instructed, and they should try to avoid eating high-cholesterol foods and eat more fruits and vegetables, to promote intestinal motility, reduce abdominal pressure, and to prevent constipation leading to increased abdominal pressure. If the patient has lower limb pain after surgery, ultrasound examination should be carried out in time. After surgery, the patient should be guided to exercise appropriately. Within 6 h after surgery, the nurse can give passive exercise and carry out hot compress and massage on the lower limb of the patient; 6 h after surgery, the patient can carry out active exercise, and they can guide the patient to carry out lower limb knee movement, deep breathing, chest expansion, and other sports to promote blood flow; one day after surgery, on the basis of the abovementioned exercises, straight leg elevation exercise of both lower limbs can be added to ensure the normal venous return of lower limbs and prevent the formation of DVT. Medical staff should patiently explain to patients and their families the hazards of DVT and the importance of various measures in order to obtain better cooperation and increase compliance.

## 5. Conclusions

The occurrence of DVT in patients after lumbar internal fixation is related to age, BMI, and time in bed. Getting out of bed in time for functional exercises after surgery can effectively prevent the formation of DVT. During the perioperative period, preoperative graded inspections, intraoperative interventions, postoperative limb exercises, and other preventive guidance can be carried out according to different individuals to prevent the formation of postoperative DVT.

RETRACTED

## Figures and Tables

**Figure 1:** Comparison of coagulation function before and after treatment in patients with DVT. (a) Comparison of PT levels before and after treatment; (b) comparison of APTT levels before and after treatment; (c) comparison of FIB levels before and after treatment; and (d) comparison of D-D levels before and after treatment. *Note.* Compared with before treatment, ^*∗*^*P* < 0.05.

**Figure 2:** Comparison of hemorheology before and after treatment in patients with DVT. (a) Comparison of plasma viscosity levels before and after treatment; (b) comparison of whole blood viscosity high-cut levels before and after treatment; (c) comparison of whole blood viscosity low-cut levels before and after treatment; and (d) comparison of hematocrit levels before and after treatment. *Note.* Compared with before treatment, ^*∗*^*P* < 0.05.

**Table 1:** Single-factor analysis of DVT in patients after lumbar internal fixation.

Factors	*n*	DVT group (*n* = 14)	Normal group (*n* = 234)	*χ* ^2^	*P*
Gender				0.062	0.803
Male	132	7(50.00)	125(53.42)		
Female	116	7(50.00)	109(46.58)		
Age (years)				6.071	0.048
<56	49	1(7.14)	48(20.51)		
56∼65	114	4(28.57)	110(47.01)		
>65	85	9(64.29)	76(32.48)		
BMI (kg/m^2^)				8.691	0.034
<18.5	54	1(7.14)	53(22.65)		
18.5∼23.9	120	4(28.57)	116(49.57)		
24∼27.9	52	6(42.86)	46(19.66)		
>28	22	3(21.43)	19(8.12)		
Smoke or not				0.411	0.522
Yes	70	5(35.71)	65(27.78)		
No	178	9(64.29)	169(72.22)		
Drinking alcohol or not				0.101	0.751
Yes	62	4(28.57)	58(24.79)		
No	186	10(71.43)	176(75.21)		
With hypertension or not				0.015	0.903
Yes	50	3(21.43)	47(20.09)		
No	198	11(78.57)	187(79.91)		
With diabetes or not				1.082	0.298
Yes	31	3(21.43)	28(11.97)		
No	217	11(78.57)	206(88.03)		
With hyperlipidemia or not				1.306	0.253
Yes	43	4(28.57)	39(16.67)		
No	205	10(71.43)	195(83.33)		
Intraoperative blood transfusion				4.902	0.027
Yes	76	8(57.14)	68(29.06)		
No	172	6(42.86)	166(70.94)		
Operation time (h)				7.226	0.027
<2	58	1(7.14)	57(24.36)		
2∼3	110	4(28.57)	106(45.30)		
>3	80	9(64.29)	71(30.34)		
Bed time (d)				10.946	0.004
<3	62	0(0.00)	62(26.50)		
3∼5	104	4(28.57)	100(42.73)		
>5	82	10(71.43)	72(30.77)		

**Table 2:** Assignment for multivariate analysis of factors.

Factors	Variable	Assignment
Age	*X*1	<56 = 0, 56∼65 = 1, >65 = 2
BMI	*X*2	<18.5 = 0, 18.5∼23.9 = 1, 24∼27.9 = 2, >28 = 3
Intraoperative blood transfusion	*X*3	No = 0, yes = 1
Operation time	*X*4	<2=0, 2∼3=1, >3 = 2
Bed time	*X*5	<3=0, 3∼5=1, >5 = 2

**Table 3:** Multifactor analysis of DVT in patients after lumbar internal fixation.

Variables	*B*	SE	Walds	*P*	OR	95%CI
Age	0.912	0.533	4.394	0.043	2.489	1.384∼3.652
BMI	0.348	0.182	5.184	0.024	1.416	1.059∼2.018
Intraoperative blood transfusion	0.147	0.224	2.158	0.172	1.158	0.689∼1.782
Operation time	0.218	0.159	1.862	0.215	1.244	0.894∼1.631
Bed time	1.215	0.684	6.125	0.011	3.371	1.941∼5.063

RETRACTED

## Data Availability

The data can be obtained from the author upon reasonable request.
